# Biomechanical Analysis of Volleyball Players' Spike Swing Based on Deep Learning

**DOI:** 10.1155/2022/4797273

**Published:** 2022-08-04

**Authors:** Lejun Hu, Kai Zhao, Wei Jiang

**Affiliations:** ^1^Zhejiang Sci-Tech University, Hangzhou 310000, Zhejiang, China; ^2^China Volleyball College, Beijing Sport University, Beijing 100089, China

## Abstract

Deep learning is to learn the inherent laws and representation levels of sample data. The information obtained during these learning processes is of great help in the interpretation of data such as text, images, and sounds. Through the deep learning method, the image features are learned independently, and feature extraction is realized, which greatly simplifies the feature extraction process. It uses deep learning technology to capture the motion of volleyball players and realizes the recognition and classification of motion types in the data. It finds the characteristics and deficiencies of the current volleyball players' spiking skills by comparing the test data of 8 volleyball players' spiking skills and biological analysis. The results show that the front and rear spiking balls with double-arm preswing technology have very obvious technical differences. In the take-off stage, there was no significant difference in the buffering time, the kick-off time, and the take-off time in the front and rear row spikes of the A-type. The buffer time of the B-type spike is 0.26 s in the front row and 0.44 s in the rear row. The range of motion of the front row spike is greater than the range of motion of the back row spike. In the air hitting stage, the range of action of the back row spiking is larger than that of the front row spiking, but the range of action of the back row is greater than that of the front row spiking.

## 1. Introduction

Over time, volleyball has become increasingly recognized by the public. Through continuous reform and improvement, it has become a world-class sport. At the same time, it is also an advantageous competitive sport in China. The Chinese women's volleyball team won five consecutive championships in 1980, and the men's volleyball team also won the fifth place in the world. However, the level of competition declined in 1990 for various reasons. Volleyball is a game played by two equal teams on an evenly divided court. The pitches are separated by nets. According to the rules of volleyball, the ball enters the opponent's court from any part of the body, but does not fall on the opponent's court in a combined offensive and defensive game. Along with football and basketball, volleyball is one of the three major sports in the world. In recent years, human action recognition, as an important branch of computer vision, is basically the correct classification of human action information in sports videos, which can be applied to the analysis process of volleyball players' spiking techniques.

Spike is one of the basic skills of volleyball. It is a method of jumping into the air and forcing the ball over the edge of the net. It is one of the most offensive techniques in volleyball and it plays an important role in the game. Spike is the main tool for scoring and the key to victory. A volleyball team's attack power is largely determined by the success or failure of the spike. Not only does hitting the ball lower the opponent's morale and cause severe psychological stress, it also enhances team spirit. However, traditional image extraction and recognition methods need to rely on experience to manually extract features. Its feature error is large and the recognition effect is not ideal. Therefore, it uses deep learning to quickly identify the spiking action and further study the action structure and action characteristics of the volleyball spiking technique. This better links the other technical movements of volleyball and improves the coaching level and the training performance of the players. It has great practical application significance.

This paper makes full use of the information of human action videos and combines it with deep learning for training and testing. It improves the accuracy of recognition and realizes the recognition and classification of action types in the data. It provides accurate action data for analysis of hitting speed and time for coaches to refer to and improve the athlete's action level.

## 2. Related Work

Volleyball is one of the most important sports in the world, and many scholars have conducted related research on it. The purpose of the Hantoush study was to determine the following: (1) To assess the stability of barrier skills and some biomechanical variables of movement in volleyball. (2) To discover differences in some biomechanical variables of barrier skills of stability and movement in volleyball. He hypothesized that there were statistically significant differences in the values of some biomechanical variables between volleyball stability and athletic obstacle wall skills. He came to the following conclusions: (1) The variable velocity of body corners from the moment of maximum flexion to the moment of leaving the ground is clearly different between stable and moving obstacle walls. And it facilitates the resistance of the barrier wall to movement. (2) It is stable between maximum flexion until reaching the highest ascent. There is a significant difference in the variable motor kinetic energy motion of the resistance wall. However, this is not very practical [1]. The purpose of the Karali et al. study was to determine predictions of quantitative athletic ability in young volleyball players based on some basic anthropological characteristics. Participants were tested for 5 morphological variables, namely, maximum spiking stretch (MSR), maximum standing block stretch (MSBR), maximum running block stretch (MRBR), ball throwing 2 kg (MEDT2KG), and 1 flexibility test - bench press forward bend (FBB). He found an obvious relationship between the variables of “maximum spike distance” (MSR), “maximum standing barrier distance” (MSBR), and “maximum running barrier distance” (MRBR) and a system of variables related to quantitative motor skills (*R* = 0.871). There was no significant relationship between ball throwing 2 kg (MEDT2KG) (*R* = 0.552) and table top bend (BFB) and the quantitative exercise capacity variable system (*R* = 0.27) [2]. Biomechanical analysis is an important direction to study the skill parameters of ball players. Peng and Tang combined deep learning (DL) technology with tennis player's shot angle selection to provide an intelligent basis for the player's biomechanical analysis. This work collects image data of tennis players using an Internet of things (IoT) Modbus-based (serial communication protocol) sensor image acquisition circuit. He used a feature map-optimized general adversarial network (GAN) to optimize video images of tennis players, and he used the VICON system to analyze joint motion metrics at different hitting angles. The results showed that the knee joint motion speeds under the two hitting angles were 2.59 ± 0.07 m/s and 2.21 ± 0.065 m/s, respectively, with significant differences (*P* < 0.05). There was a significant difference in the speed of the right ankle and right hip in the swing phase of forehand topspin and forehand flat spin (*P* < 0.05) [3]. The main purpose of Hongtao's research was to perform a biomechanical analysis of dunk techniques, especially the analysis of bounce force and stamina when dunking. He employed the method of non-Cybex combined with multijoint velocity measurement and motion video recording. He also conducted a biomechanical analysis of the equivalent strength of the standing long jump, step jump, and spring force. Combined with the analysis and research of air volleyball technology, it can study the mechanics of softball [4]. The purpose of the Rusdiana study was to use a portable smart platform with Android Pi to analyze the kinetic and kinematic parameters of the starting motion in swimming for the application of sports biomechanics. These results demonstrate a high degree of stability using prototypes and commercial products. The prototype he developed can be used as a surrogate to measure maximum leg strength, reaction time, and ground response at the start of swimming. The product has the advantages of low cost, portability, and real-time performance [5]. Nei et al. researched important training methods for improving the tactics of youth volleyball players. In practice, coaches quickly move from learning the 6 : 0 system (initial system) to the 5 : 1 system (competitive-advanced). For beginners, this results in limited performance of tactical and strategic skills. This also affects the effectiveness of technical elements in the game. The purpose of this article is to demonstrate an age-oriented and time- and experience-oriented systematic approach to volleyball learning. Order in training, respect for age, sport and sporting age, timely specialization, and principles of sport-oriented learning are identified as factors that lead to expected outcomes in an individual athlete's career. This makes the training method effective and desirable in practice [6]. Freehand pitching is a movement that requires coordination of the lower body, trunk, and upper body to effectively transfer force throughout the kinematic chain to throw a baseball. The purpose of the Rusdiana et al. study was to investigate the effect of cardiorespiratory fatigue on pitching speed in relation to changes in baseball kinematic movement. Cardiorespiratory fatigue leads to changes in the coordination of movements of the upper and lower extremities, which can lead to a decrease in ball speed. These results are similar to those of a previous study of an intervention on muscle fatigue during high altitude baseball throwing, which resulted in a decrease in performance and ball speed [7]. These methods provide some references for the research, but due to the short time and small sample size of the relevant research, this research has not been recognized by the public. However, there are relatively few studies on the biomechanical analysis of volleyball players' spike swings based on deep learning techniques. It is necessary to fully apply these techniques to research in this field.

## 3. Combination Method of Volleyball Player Spiking and Arm Swing Based on Deep Learning

### 3.1. The Development of Volleyball

Volleyball is a collective sport, with offensive and defensive confrontation as the main means, emphasizing the comprehensiveness of offensive and defensive techniques, and paying attention to the play at the overall technical and tactical level. The basic skills of volleyball mainly include offensive and defensive skills [8]. Among them, offense is an important guarantee for winning the game, and spiking is the core means of offense. Looking at the volleyball world in today's world, due to the different physical conditions and development concepts, the technical schools of volleyball show diverse characteristics. There are not only European power factions represented by Russia, Serbia, etc., but also technical factions represented by Brazil, the United States, and China, and defensive counterattacks represented by Japan [9]. According to its power characteristics, the smash can be divided into strong smashes, light smash, and lob.

The technical structure and movement mechanism of different spiking types are different. Among them, the technical structure and movement mechanism of vigorously spiking are the most complicated. The light smash technique is relatively simple, easy to learn, and easy to master. It has the characteristics of strong suddenness, small error rate, and easy scoring. People with volleyball foundation can basically use [10]. In particular, young people have technical shortcomings such as slow foot movement and poor defensive judgment due to physical limitations during the game. The use of light spiking technology will effectively make up for the lack of technology, which is of great help in winning the game. The process diagram of the action process of the spiking technique is shown in Figure 1 [11].

Aerial shot is an action done in the air when the body loses its support point. The human body swings arms and hits the ball in the air mainly by relying on the strength of the body itself. The spiking action is a “beating whip” action. The whiplash action is that the large joint drives the small joints, and the large and small joints move in sequence [12]. The velocity of the end of the arm (the palm of the hand) is formed by the sequential transfer of the momentum of the proximal link and the superposition of the velocity. Modern professional volleyball tends to be increasingly intense confrontations with high intensity, high difficulty, and high skill. Therefore, it is a very effective measure to use advanced science and technology to improve the level of Chinese volleyball and accurately obtain and analyze the sports data of athletes in detail [13].

### 3.2. Deep Learning Theory

Deep learning technology has developed with the development of computer hardware technology, cloud computing, and big data technology. It is based on an artificial neural network [14]. Its emergence has led to the rapid development of fields such as speech recognition, image processing, and natural language processing. Deep learning is a broad class of machine learning techniques and architectures. It is characterized using some nonlinear hierarchical information processing. According to different application fields and network structures, network architectures can be divided into three categories:

1. Unsupervised deep learning network. It is used for learning without class label information. This approach is similar to a clustering algorithm. It can automatically acquire class labels through subsequent learning [15];
2. Supervised deep learning network. It directly discriminates the category according to its own discriminative ability, and describes the posterior distribution of the category under the condition of visible data;
3. Hybrid system deep learning network. By combining 1 and 2 to obtain more accurate discriminative results, the hybrid system deep learning network still belongs to the discriminative model [16].

According to the three types of structures mentioned above, this paper classifies the commonly used network models. In the broad category of unsupervised deep learning networks, effective samples are generated by learning data from the network and collecting samples [17]. Such network models include restricted Boltzmann machines, deep belief networks, deep Boltzmann machines, generalized denoising autoencoders, and recurrent neural networks. In supervised deep learning networks, there are mainly LSTM network models and neural network models such as CNN. The hybrid system deep learning network mainly includes the combination model of the deep belief network and the deep neural network, and the new combination model of the deep belief network and the Markov model [18].

Although the motion energy map can reflect the spatial information of the action, it cannot reflect its temporal information [19]. It sets *D* as the intensity value of the motion history pixel and *D*_*τ*_(*x*, *y*, *t*) as the update function, which can be calculated as follows:

(1) $$\begin{array}{c} D_{\tau }\left(x,y,t\right)=\tau ,\text{if }\varphi \left(x,y,t\right)=1,\\ D_{\tau }\left(x,y,t\right)=\max\left(0,D_{\tau }\left(x,y,t-1\right)-\gamma \right).\;\text{otherwise.} \end{array}$$

In the above formula, (*x*, *y*) represents the position of the pixel, and *t* is the time; *τ* is the duration, which defines the relationship between the time interval of the motion and the number of frames; *γ* is the elapsed parameter [20]. The update function *D*_*τ*_(*x*, *y*, *t*) can be determined by several methods, such as optical flow, frame difference, and image difference. The principle of the frame difference method is to use pixel-based time difference between two adjacent frames or three frames of the image sequence to extract the moving area in the image through closing values. The frame difference method is the most commonly used, and its application is shown in the following formula:

(2) $$\begin{array}{c} \varphi \left(x,y,t\right)=1,\text{if }S\left(x,y,t\right)\geq \lambda ,\\ \varphi \left(x,y,t\right)=0.\;\text{otherwise.} \end{array}$$

In

(3) $$\begin{array}{c} S\left(x,y,t\right)=\left|V\left(x,y,t\right)-V\left(x,y,t\pm \Delta \right)\right|. \end{array}$$

Among them, *V*(*x*, *y*, *t*) represents the intensity value of the pixel whose coordinate is in the *t*-th frame of the video image sequence, (*x*, *y*) is the distance between frames, and Δ is an artificial difference threshold. They can be adjusted as the video scene changes [21].

The most widely used deep learning networks in image processing are deep belief networks and convolutional neural networks [22].

#### 3.2.1. Deep Belief Network

A deep belief network model is a probabilistic generative model that contains multiple hidden layers to generate the most likely data by training the weights of neurons in the hidden layers. The neurons in each layer are independent of each other, and two adjacent hidden layers in the network are combined by a restricted Boltzmann machine (RBM) [23].

As shown in Figure 2, a deep belief network consists of six layers. The deep belief network uses a deep learning network model that composes of an input layer *I*, an output layer *O*, and *n* hidden layers in series. We combine all RBMs with unsupervised learning methods to form a deep trust network model. DBN can use a common probability density distribution to represent the relationship between the input layer and the hidden layer. It assumes that the DBN contains *n* hidden layers and *x* is the input data. The joint probability density distribution is as follows:

(4) $$\begin{array}{c} P\left(x,h^{2},h^{3},\ldots ,h^{n}\right)=\prod_{c=1}^{n-2}P\left(h^{c}|h^{c+2}\right)P\left(h^{n-2}|h^{n}\right). \end{array}$$

In the formula, *x*=*h*^0^ and *P*(*h*^*c*^*|h*^*c*+2^) are conditional probability distributions.

For values in a visible or hidden layer, values from other layers do not affect each other.

(5) $$\begin{array}{c} P\left(h|r\right)=\prod_{j=1}^{M}P\left(h_{j}|r\right), \end{array}$$

or

(6) $$\begin{array}{c} P\left(r|h\right)=\prod_{i=1}^{N}P\left(r_{i}|h\right), \end{array}$$

where *M* is the number of neurons in the visible layer and *N* is the number of neurons in the hidden layer. It assumes that the input data of the visible layer is *x* and the output data of the hidden layer is *h*. The energy function *E*(*x*, *h*) is:

(7) $$\begin{array}{c} E\left(x,h\right)=-\sum_{i=1}^{M}A_{i}x_{i}-\sum_{j=1}^{N}B_{j}x_{j}-\sum_{i=1,j=1}^{M,N}h_{j}x_{i}k_{ij}, \end{array}$$

where *A* and *B* are the biases of the visible and hidden layers, respectively. *K* represents the weight. The joint probability between *x* and *h* is

(8) $$\begin{array}{c} P\left(x,h\right)=\frac{1}{G}e^{-E\left(x,h\right)}, \end{array}$$

where *G* is the normalization factor whose value is

(9) $$\begin{array}{c} G=\sum_{x,h}e^{-E\left(x,h\right)}. \end{array}$$

Also, the probability distribution function about the occurrence of the *x* state is

(10) $$\begin{array}{c} P\left(x\right)=\sum_{h}P\left(x,h\right)=\sum_{h}\frac{e^{-E\left(x,h\right)}}{G}. \end{array}$$

It assumes an intermediate variable *f*(*x*) as

(11) $$\begin{array}{c} f\left(x\right)=-\log\sum_{h}e^{-E\left(x,h\right)}. \end{array}$$

Then,

(12) $$\begin{array}{c} P\left(x\right)=\frac{e^{-f\left(x\right)}}{G},\\ G=\sum_{x,h}e^{-f\left(x\right)}. \end{array}$$

It can be seen from the above formula that the RBM can enter a stable state only when *f*(*x*) is the smallest, that is, when *P*(*x*) is the largest and the energy value is the smallest.

#### 3.2.2. Convolutional Neural Network

A convolutional neural network is a deep learning network with multiple layers of neurons. It is widely used in image processing because it can be used directly on image data without extensive and complex preprocessing. It extracts features from images using successive convolution and clustering layers, and finally uses a fully connected layer for label classification. Convolutional neural networks use local connection strategies and weight distribution strategies and subsampling functions to further reduce parameters. In the idea of local connection, neurons only need to process local parts, and then the next level organizes this local information into global information.  Figure 3 shows a common structure of convolutional neural networks. It has no explicit requirements for the order of convolution and pooling. It can continue the convolution operation after the first convolution layer and can also perform pooling.

As shown in Figure 3, convolutional neural networks are computationally intensive and require high computing power of computing devices. Only using the central processing unit in the computer cannot effectively speed up the calculation, and most methods will use a general-purpose image processor to speed up the processing of data. The idea of local connection is based on the fact that the image data is tightly connected locally and weakly connected in the distance, which also expresses complete information. Subsampling is mainly used for pooling layers. Subsampling uses max or average samples to handle the very large parameters produced by convolutional layers. It assumes that the sample size is *n* × *n* and the sample parameter dimension becomes 1/*n*^2^. This greatly reduces the dimension of parameters and effectively reduces the parameter overfitting. The expression for the pooling layer is given by the following relation:

(13) $$\begin{array}{c} W_{j}^{i}=f\left(w_{j}^{i}\cdot \text{down}\left(x_{j}^{x-1}\right)\right)+d_{j}^{i}, \end{array}$$

where down(·) in the formula is the subsampling operation. *w*, *d* are the weights and biases, respectively.

Neurons are the basic elements of convolutional neural networks, and their structure is shown in Figure 4. *x*_1_, *x*_2_,…, *x*_*n*_ is the *n* inputs in the graph, and *w*_*i*,*j*_ represents the corresponding input weight. Here, *i*=1,…, *n* , *θ* is the activation threshold and *f*(·) is the activation function of the neuron. Then the output data of the *j*th neuron *Y*_*j*_ can be defined as follows:

(14) $$\begin{array}{c} Y_{j}=f\left(\sum_{i=1}^{n}w_{i,j}x_{i}-\theta_{j}\right). \end{array}$$

## 4. Experiment of Volleyball Player's Spiking Arm Swing Based on Deep Learning

For the volleyball spiking technique, different players have their own characteristics. Different players use different techniques to a certain extent for the same position and the same type of spike. This paper studies the frontal spiking in volleyball spiking, including the front row attack of No. 4 and the back row of No. 6. Through experimental observation and data analysis and screening of video analysis, the technical movements of the subjects in this experiment are divided into two types in the take-off stage based on the differences in the take-off techniques of the subjects. It defines them as “Type A” and “Type B.”

“Type A” with a total of 7 people, accounting for 88% of the subjects. It takes the right arm smash player as an example. In the last step of the approach, the athlete takes a big step with his right foot first, and then his left foot quickly joins. When the athlete steps out with his right foot, he pulls his arms backward and upward through the side of the body. Their left foot and up to the braking process, and the arms swing forward actively from the back. They jumped upwards with their legs slammed on the ground, and their arms also swayed upwards to match the take-off. This type of take-off technique has a large range of swing arm movements, obvious pull-back of the arms, and obvious characteristics of the front and rear spiking take-off, which is a common technique.

“Type B” with only one person, accounting for 12% of the subjects. It takes the right arm smash player as an example. In the last step of the approach run, the athlete takes a big step with the right foot first, and the right leg brakes and cushions. They then moved up slowly to their left foot, before the right foot, keeping their arms by their sides with little to no swing. They jumped upwards with their legs slammed on the ground, and their arms swayed upwards with force to take off. In this type of take-off technique, the swinging arm movement range is small, the arms are basically not drawn back, and the lower limbs are fully buffered. However, the characteristics of the front and rear spikes are not obvious, which is a special technique.

Before the experiment, the basic information data of the 8 players selected by the experimental group were statistically analyzed, and different experimental subjects were represented by numbers. As shown in Table 1.

This experiment focuses on the spiking action of volleyball. In the experiment, two (powerful offense from 4 and strong offense of 6 from the back row) representative actions were selected for comparative analysis. It focuses on the kinematic parameters of the four take-off stages from take-off to midair bounce. The kinematics testing instruments include 2 domestic high-speed cameras, 2 notebooks, 1 set of 3D frames, 3 full lights (because the experiment is carried out indoors, the images collected by high-speed cameras are dark and unclear, and a fill light is needed to improve the brightness), 6 tripods, and several data cables. It uses the three-dimensional high-speed camera test to shoot the whole body of the subjects from the take-off stage to the air hitting stage of the front and rear row of the attacking smash. The data acquisition and processing process of the experimental object is shown in Figure 5.

## 5. Biomechanical Analysis of Volleyball Players Spiking and Swinging

### 5.1. Results and Analysis of the Take-Off Stage

Table 2 shows the time used in the buffer stage and the kick-off stage of the front and rear spikes of “Type A” and “Type B.”

Through the study of various influencing factors on volleyball spiking technical movements, it is concluded that among various influencing factors, the time structure factor has the greatest influence. Time is the parameter with the largest contribution rate. The table shows the time used in the buffer stage and the kick-off stage of the “A-type” and “B-type” front and rear spikes. In the A-type front and rear spiking segment, there was no significant difference in landing time, kicking time, and total take-off time between front and rear spiking. However, whether it is the front row spiking or rear row spiking, the buffering time is less than the kicking and extension time. In the B-type front and rear row spikes, the buffer time of the front row spikes was shorter than that of the rear row spikes, and there was no significant difference in the kick-off time. This shows that the cushioning is more adequate when spiking the ball in the back row.

### 5.2. Results and Analysis of the Flight Stage

There are two stages in the aerial shot link: the back swing stage of the spike arm and the front swing stage of the spike arm. If the process of hitting the ball in the air is regarded as archery by drawing a bow, then the back swing phase of the spiking arm is equivalent to the process of drawing the bow full of strings, and the front swing phase is the process of shooting arrows with a string.  Figure 6 lists the time indicators of the flying shot, including the time from jumping to hitting, arm time, and arm swing time.

From the analysis of the front and rear spikes, the paired sample *t*-test shows that the arm swing time of Type A is significantly different (*p* < 0.01), indicating that the process of finding the ball and hitting the ball is long, and the time from jumping to hitting the ball is significantly different. There was no difference in pull-up time (*p* > 0.05). The B-type has basically no difference in the comparison of front and rear spikes, which has a lot to do with the type of technology. This type of technology is basically the same in the front and rear in the run-up and take-off technology, so the movements in the air also have the same characteristics.

From the comparative analysis of different types of techniques, it can be seen that there is basically no difference between A and B in the time from take-off to hitting, while the B-type technique has longer bow arm time and shorter arm swing time. This shows that the B-type technology has a larger range of action when the arm is pulled up, and the arm swing time is shorter, which means that the explosion is stronger, and the momentum transfer of the spiking arm is faster.

Figure 7 is a comparison of volleyball players' arm swing time and the speed of the shoulder, elbow, and finger-metacarpal joints at the moment of hitting the ball.

Figure 8 is the upper limb speed-time curve in the front row and rear row spiking forward swing stage of Type A.  Figure 9 is the upper limb speed-time curve in the front and rear spiking stages of the B-type.

Observing Figures 8 and 9, it can be seen that whether it is Type A or Type B, whether it is a front row spiking or a back row spiking, there are consistent laws in these four speed-time curves. The shoulder and elbow curves are first rising and then falling, while the wrist and fingertip curves are first falling and then rising. The peaks of each curve appear in chronological order. The order of appearance from early to late is shoulder, elbow, wrist, and fingertips. The changing process of the four curves illustrates the speed transfer process. This is completely in line with the principle of arm whipping action when smashing the ball. The acceleration of the shoulder joint drives the movement of the elbow joint, and the acceleration of the elbow joint promotes the movement of the wrist joint. Acceleration of the wrist joint facilitates movement of the fingertip joints. In this process, the momentum is transmitted sequentially through the shoulder, elbow, wrist, and fingertips. The velocity of the ligament increases as the mass of the ligament decreases as energy is sequentially transferred from the large joint to the facet joint, which reaches its maximum velocity at the fingertips.

### 5.3. Angle Index of Arm Swing Stage

The joint angles in Table 3 refer to the joint angles at the moment when the ball rebounds strongly after being hit. Players 2, 6, and 8 are on the left side of the batter, and the rest are on the right. It can be seen from the table that No. 2 players have the largest shoulder rotation angle at the moment of hitting the ball, while No. 1 and No. 3 have smaller shoulder rotation angles below 30°. There was no significant difference in the hip and elbow joint angles of the eight players at the moment of impact. Players 2, 6, and 8 had less shoulder rotation than the other seven players.

The front and rear row spikes with A-type technology have similar movement technical characteristics as a whole. Its movement from jumping to hitting each link of the body conforms to the sequence of human joint activities. There are also differences in details compared with the front row spiking and back row spiking. In the take-off link, the front row spiking is more fully buffered, while the rear row spiking is not as good as the front row to reduce the loss of horizontal speed and momentum. Comparing the two technologies of spiking A and B, the technical characteristics of the front and rear row of the A-type technology are clearly different, and the technical characteristics of the front-row spiking of the B-type technology are basically the same, and the technical characteristics of the front-row spiking of the type-A technology are similar. In addition to the swing range of the arms during the buffering stage, whether it is the front row spiking or back row spiking, the technique has the characteristics of a large range of movements and a long movement time.

## 6. Conclusion

Spike is the most aggressive technique in volleyball and plays an important role in the game. Based on the achievements of deep learning in the field of human motion, this paper conducts an in-depth study of the principles of deep learning. It studies the technical activities of volleyball players' spiking and swinging arms and obtains the kinematic parameters of volleyball players' technical characteristics. There are many obvious differences in the technical characteristics of front and rear spikes with double arms with preswing technology. During the starting phase, the front row spikes have a greater range of motion than the back row. During the aerial shot phase, the range of motion of the rear spike is greater than that of the front peak. The hands have a rhythm of muscle activity before swinging. Throughout exercise, muscle activity throughout the body is balanced. The contribution of each muscle is equal, and the primary and secondary ratio of muscle strength is not obvious. Only by combining the speed and timing of the shot, and the biological principles of the hitting action to form thebest hitting point, can the athlete have room for improvement.

## Figures and Tables

**Figure 1:** Schematic diagram of the spiking action process.

**Figure 2:** Deep belief network model.

**Figure 3:** Convolutional neural network architecture.

**Figure 4:** Neuron structure diagram.

**Figure 5:** Data acquisition and processing of experimental subjects.

**Figure 6:** Time for each stage of airing.

**Figure 7:** Comparison of volleyball players' arm swing time and shoulder, elbow, and finger-to-metacarpal joint speeds at the moment of hitting the ball.

**Figure 8:** The upper body speed-time curve during the front and rear spikes of Type A.

**Figure 9:** The upper body speed-time curve in the front and rear spiking phases of the B-type.

**Table 1:** Registration form of basic information of subjects.

Athlete number	Height (cm)	Body weight (kg)	Age (year)	Campaign level	Position on the field	Arm buckle
1	1.95	76	22	Level 1	Main attack	Right
2	1.93	78	23	Level 1	Main attack	Left
3	1.90	84	23	Level 1	Secondary attack	Right
4	1.96	100	23	Level 1	Stand ready for assistance	Right
5	1.94	94	24	Level 1	Free man	Right
6	1.97	86	25	Level 1	Secondary attack	Left
7	1.96	85	23	Level 2	Main attack	Right
8	1.95	87	25	Level 2	Second pass	Left

**Table 2:** Time of each stage of take-off (unit: s; Type A, *n* = 7; Type B: *n* = 1).

Parameters	Type A front row	Type A rear row	Type B front row	Type B rear row
	$\bar{x}\pm S$	$\bar{x}\pm S$		
Landing buffer time	0.15 ± 0.02	0.16 ± 0.03	0.26	0.44
Stirrup extension off the ground time	0.21 ± 0.01	0.23 ± 0.02	0.30	0.30
Take off time	0.36 ± 0.03	0.39 ± 0.05	0.56	0.74

**Table 3:** Angle indicators of body-related joints at the moment of hitting the ball in the swing stage.

Athlete number	Shoulder spin angle at the moment of hitting the ball (°)	Hip joint angle (°)	Elbow joint angle (°)	Shoulder joint angle (°)
1	26.31	157.58	144.87	156.24
2	64.56	153.24	143.62	139.62
3	28.61	160.32	135.62	165.55
4	37.84	169.35	146.95	160.24
5	42.85	165.27	151.24	152.84
6	63.59	155.24	143.55	139.62
7	55.62	170.24	152.34	140.24
8	64.55	153.85	144.20	139.84

## Data Availability

Data sharing not applicable to this article as no datasets were generated or analysed during the current study.
